The article "Dynamic Enhanced Magnetic Resonance Imaging versus Ultrasonic Diffused Optical Tomography in Early Diagnosis of Breast Cancer" was retracted in 2023. Reason: concerns about the peer review.

# Dynamic Enhanced Magnetic Resonance Imaging versus Ultrasonic Diffused Optical Tomography in Early Diagnosis of Breast Cancer

**DOI:** 10.1155/2022/4834594

**Published:** 2022-04-12

**Authors:** Feng Xue, Jie Jiang

**Affiliations:** ^1^Hepatobiliary Surgery, Qingdao Jiaozhou Central Hospital, Qingdao City 266300, Shandong Province, China; ^2^Radiology Department, Affiliated Hospital of Shandong University of Traditional Chinese Medicine, Jinan City 250011, Shandong Province, China

## Abstract

**Objective:**

To compare the application value of dynamic enhanced magnetic resonance imaging (MRI) and ultrasonic diffused optical tomography (DOT) in early diagnosis of breast cancer.

**Methods:**

The clinical data of 110 female patients with breast diseases treated in our hospital from June 2018 to June 2021 were selected for the retrospective analysis, and the patients were divided into the benign lesion group (*n* = 50) and breast cancer group (*n* = 60) according to the pathologic findings. All patients received dynamic enhanced MRI and ultrasonic DOT examinations for the observation of lesion morphology and analysis of relevant parameters, so as to scientifically evaluate the diagnostic value of dynamic enhanced MRI and ultrasonic DOT for early breast cancer.

**Results:**

The dynamic enhanced MRI examination found that the proportions of irregular shape, increased vascular shadow, obscure boundary, spicule sign, heterogeneous enhancement, etc. of lesion were significantly higher in the breast cancer group than in the benign lesion group (*P* < 0.05); parameters such as *K*^trans^, *K*_ep_, and *V*_*e*_ were significantly higher in the breast cancer group than in the benign lesion group (*P* < 0.05); the ultrasonic DOT diagnosis found that the THC value was obviously lower in the benign lesion group than in the breast cancer group (*P* < 0.05); compared with the pathologic findings, it was believed that combined diagnosis had significantly higher diagnosis accuracy rate, sensitivity, specificity, positive predictive value and negative predictive value than the dynamic enhanced MRI and ultrasonic DOT diagnosis alone (*P* < 0.05); and after further analyzing the efficacy of the two diagnosis modalities in diagnosing early breast cancer by ROC curves, the result showed combined diagnosis > dynamic enhanced MRI > ultrasonic DOT.

**Conclusion:**

Both dynamic enhanced MRI and ultrasonic DOT present higher diagnostic value to early breast cancer, of which dynamic enhanced MRI obtains results closer to the pathologic findings and has diagnostic efficacy higher than ultrasonic DOT. But the combination of the two can significantly improve the diagnosis accuracy rate for early breast cancer, presenting higher diagnostic value.

## 1. Introduction

According to the survey data of the International Agency for Research on Cancer (IARC) in 2018, the incidence of breast cancer ranks first among female cancers, which accounts for 24.2% of the global female cancer incidence [1]. Moreover, the incidence of breast cancer in China also shows an increasing trend year by year, and even though new treatment strategies and methods are gradually popularizing, the mortality of breast cancer in China has not lowered significantly [2, 3]. The early symptoms of breast cancer are not typical, thus palpation, serum tumor marker detection, and core needle biopsy (CNB) all show some limitations in early diagnosis[4–7]. Currently, imaging examination is still the main strategy for early diagnosis of breast cancer, and the two commonly used examination modalities are ultrasound and magnetic resonance imaging (MRI). MRI plain scan can accurately localize the lesion morphology, with the help of dynamic contrast-enhancement (DCE) method, the paramagnetic contrast medium is introduced to get the qualitative curve characteristics and quantitative parameters of contrast penetration and clearance inside the tumor, so that the pathological and physiological behavior is intuitively manifested, with the diagnostic efficacy that has been confirmed in common cancers such as cervical cancer and lung cancer [8, 9]. Ultrasonic diffused optical tomography (DOT) is a novel functional imaging system capable of reflecting the morphological information and metabolic status of breast masses to achieve the identification and diagnosis of breast cancer. From a theoretical point of view, both examination modalities can estimate the nature of masses, and they present different shortcomings in the clinical practice. There are few reports on the comparative analysis and combined application. Hence, to further clarify the features and advantages of dynamic enhanced MRI and ultrasound DOT in the diagnosis of breast cancer, 110 female patients with breast diseases treated in our hospital were selected as the study objects for the comparative analysis on application value of dynamic enhanced MRI and ultrasound DOT in early diagnosis of breast cancer, with the results reported as follows.

## 2. Materials and Methods

### 2.1. Cases Screening and Grouping

The inclusion and exclusion criteria were proposed according to the study objective. Inclusion criteria: ① All patients were diagnosed after puncture or surgical pathology; ② all patients were over 18 years old; ③ all patients could finish the dynamic enhanced MRI and ultrasonic DOT examinations; and ④ the patients and their family members signed the informed consents after fully understanding the study objective, process and value. Exclusion criteria: ① The patients had history of surgery, chemoradiotherapy or treatments for other tumors before this diagnosis; ② the patients had received breast prosthetic implantation before; ③ the patients had cognitive disorder, hearing-seeing disorder or language communication disorder; ④ the patients had surgery, puncture or MRI contraindication; ⑤ the patients had other malignant tumors; and ⑥ the patients' estimated survival was less than 6 months. The clinical data of 110 female patients with breast diseases treated in our hospital from June 2018 to June 2021 were selected for the retrospective analysis, and the patients were divided into the benign lesion group (*n* = 50) and breast cancer group (*n* = 60) according to the pathologic findings. The study met the World Medical Association Declaration of Helsinki [10].

### 2.2. Dynamic Enhanced MRI Examination

The patients were in the prone position, with both hands naturally placing on two sides of the body, and the cross-sectional T1WI and fat suppression T2WI (fs-T2WI) scanning to the bilateral breast, auxiliary and mediastinum was performed by Magnetom Verio 3.0 T MRI (manufacturer: Siemens Company, Germany) and 8-channel breast phase array coil [11–13]. T1WI: Fl3d-nonfs sequence, i.e., TR of 3.92 ms, TE of 1.39 ms, 3 mm layer thickness, 0.25 mm layer gap, 360 mm × 360 mm FOV, 384 × 288 matrix; fs-T2WI: inversion recovery sequence, i.e., TR of 550 ms, TE of 11 ms, 90° flip angle, 3 mm layer thickness, 0.5 mm layer gap, 360 mm × 360 mm FOV, 384 × 256 matrix. After scanning, contrast agent Gd-DTPA was injected with high pressure syringe (rate: 2.5 ml/s; dose: 0.1 ml/kg), and 20 ml of normal saline was injected to wash the tube (rate: 2.0 ml/s), then DCE scanning with Vibe fat suppression sequence was performed immediately with the following parameters: TR of 4.57 ms, TE of 1.57 ms, 25° flip angle, 1 mm layer thickness, 0.5 mm layer gap, 360 mm × 360 mm FOV, and 512 × 512 matrix, one image was acquired every 20 s during the first 3 min of continuous scanning, and then every 100 s during the following 10 min of continuous scanning, and all images were processed and analyzed by ADW4.4 workstation. The diagnosis was made by 1 experienced MRI diagnostic physician in radiology department by the double blind method. First, the physician observed the lesion morphology and enhancement characteristics, selected the most obvious image for enhancement to outline the region of interest (ROI) and then obtained the volume transfer constant (*K*^trans^), reverse reflux rate constant (*K*_ep_) and extracellular extravascular volume fraction (*V*_e_) images, and measured parameters including *K*^trans^, *K*_ep_ and *V*_*e*_ on the corresponding pseudo-color image.

### 2.3. Ultrasonic DOT Examination

A dual-mode imaging system composed of XinAoMDT mammary gland diagnostic apparatus (model: OPTIMUS II), ultrasonic diagnostic device (model: Terason 13000; parameter: 7–12 MHz of array probe frequency; manufacturer: Teratech USA) and DOT system was established. First, the lesion was positioned by routine ultrasound, and then optical scanning of the mammary gland in affected side was performed: the largest section of the lesion was used as the horizontal section for optical scanning, then, the probe was rotated 90 degrees for optical scanning of vertical section, and the images were saved; optical scanning was performed on mirror symmetric section of the contralateral breast versus the lesion of the affected side, and the ROI was outlined on the two lesion sections for optical reconstruction to obtain the optical characteristic parameters, THC and light absorption image [14].

### 2.4. Study Methods

All patients received puncture or surgery within two weeks after MRI examination and ultrasonic DOT examination, and pathological examination of specimens was conducted to confirm the diagnostic results.

### 2.5. Statistical Processing

In this study, the between-group differences in data were calculated by SPSS22.0, the picture drawing software was GraphPad Prism 7 (GraphPad Software, San Diego, USA), the items included were enumeration data and measurement data, which were expressed by [*n*(%)] and ($\bar{x}\pm s$) and examined by *X*^2^ test and *t*-test, respectively, and differences were considered statistically significant at *P* < 0.05.

## 3. Results

### 3.1. General Data

No statistical differences in patients' general data including age, BMI, tumor diameter, histological grade, and number of masses were observed (*P* > 0.05). See Table 1.

### 3.2. Dynamic Enhanced MRI

The dynamic enhanced MRI examination found that the proportions of irregular shape, increased vascular shadow, obscure boundary, spicule sign, heterogeneous enhancement, etc. of lesion were significantly higher in the breast cancer group than in the benign lesion group (*P* < 0.05); and parameters such as *K*^trans^, *K*_ep_, and *V*_*e*_ were significantly higher in the breast cancer group than in the benign lesion group (*P* < 0.05). See Tables 2 and 3.

### 3.3. Ultrasonic DOT

According to Table 4, ultrasonic DOT diagnosis found that the THC value was obviously lower in the benign lesion group than in the breast cancer group (*P* < 0.05), with statistically significant difference.

### 3.4. Comparison of Diagnostic Results of Dynamic Enhanced MRI and Ultrasonic DOT

According to the statistical results in Tables 5 and 6, compared with the pathologic findings, it was believed that combined diagnosis had significantly higher diagnosis accuracy rate, sensitivity, specificity, positive predictive value (PPV) and negative predictive value (NPV) than the dynamic enhanced MRI and ultrasound DOT diagnosis alone (*P* < 0.05).

### 3.5. Diagnostic Efficacy Analysis

After further analyzing the efficacy of the two diagnosis modalities for diagnosing early breast cancer by ROC curves (see Figure 1 and Table 7), the result was combined diagnosis > dynamic enhanced MRI > ultrasonic DOT.

Sig. referred to the *P* value, when the corresponding value of sig. was less than 0.05 (significance level), it indicated that the regression equation was statistically significant, that is, there was a linear relationship between the independent and dependent variables.

## 4. Discussion

### 4.1. Diagnostic Value of Ultrasonic DOT in Early Breast Cancer

An important step in tumor cell growth and metastasis is the formation of new blood vessels, and malignant tumors are able to further stimulate the production of new capillaries with angiogenic growth factors, which in turn increase local blood volume and hemoglobin content to meet the growing and metabolic demands of tumor cells [15, 16]. Therefore, cancer cells are metabolically exuberant with increased oxygen consumption, which gives malignant tumor cells the peculiar phenomenon of “high blood and low oxygen” inside; with less new blood vessels in benign tumor cells, the oxyhemoglobin and deoxyhemoglobin inside the tumor are close to the surrounding normal tissue [17, 18]. Thus, with presentation of the diffused optical image of the lesion site according to the optical signal and combination with the anatomical information provided by ultrasound, ultrasonic DOT is able to judge the vascularity and oxygenation status within tissues by measuring the hemoglobin and deoxyhemoglobin contents, and then provides an information basis for the early diagnosis and identification of breast cancer. In this study, ultrasonic DOT diagnostic results showed that the THC value was obviously lower in the benign lesion group than in the breast cancer group (*P* < 0.05), and according to the comparison with pathologic findings, ultrasonic DOT diagnosis obtained an accuracy rate of 80.91%, sensitivity of 83.33%, specificity of 78%, PPV of 91.97%, and NPV of 79.59%, which was consistent with the report by Makela and Foster [11] further proving the higher application value of ultrasonic DOT in diagnosing early breast cancer. Ultrasonic DOT uses the parameters of high blood and low oxygen indexes of near-infrared light as the qualitative diagnostic criteria for breast cancer, which is compatible with the blood supply characteristics of most breast cancer tissues, thus it has high feasibility in diagnosing breast cancer, can complete the quantitative determination of the functional indicators within tissues and determine the tissue functionality, which are unachievable by other imaging modalities.

### 4.2. Diagnostic Value of Dynamic Enhanced MRI in Early Breast Cancer

The high spatial resolution and contrast of MRI for soft tissues are also superior to other imaging tests, and dynamic enhanced MRI can detect tiny and multiple lesions that are not easily visualized while not being affected by the degree of density of glandular tissue, which provides lesion information by establishing structural relationships of morphology, boundaries, signal intensity with surrounding tissues. Shalin et al. [19] reported that for advanced or end-stage breast cancer, MRI image can clearly determine the metastasis of lymph nodes and the invasion of lesions into the chest wall, nipples, and ribs, and has a positive guiding value for prognosis prediction. Because there is heterogeneity in the growth of cancer cells and their stroma toward the periphery, and the degree of invasion tends to be different in different directions, cancer cells often show heterogeneous morphology and margins. In this study, the dynamic enhanced MRI examination found that the proportions of irregular shape, increased vascular shadow, obscure boundary, spicule sign, heterogeneous enhancement, etc. of lesion were significantly higher in the breast cancer group than in the benign lesion group (*P* < 0.05), which confirmed the more uniform distribution of tumor morphology and margin characteristics in benign tumors than in malignant tumors, demonstrating the specificity in breast cancer lesion morphology. However, previous studies pointed out that with the increase of early examined cases, a certain proportion of cancer cell lesions with uneven growth do not fully reflect the gross morphology, so the possibility of breast caner cannot be excluded by typical round-like morphology and smooth margin characteristics.

Tumor tissue has a good environment of blood flow supply to meet its efficient energy metabolism and supply and provide nutrition delivery, immune regulation inhibition, metabolite exclusion and cytokine secretion, and therefore, the state of angiogenesis often determines the malignant biological behaviors such as tumor growth, infiltration and metastasis [20, 21]. Dynamic enhancement technology enables the analysis of functional information such as cellular composition, vascular permeability, interstitial pressure, blood flow supply, and extracellular space from a hemodynamic perspective through the dynamic distribution process of contrast agent inside the tumor [22–24]. It was concluded herein that dynamic enhanced MRI parameters such as *K*^trans^, *K*_ep_ and *V*_*e*_ were significantly higher in the breast cancer group than in the benign lesion group (*P* < 0.05), indicating that *K*^trans^, *K*_ep,_ and *V*_*e*_ could provide a strong reference for early diagnosis of breast cancer. Dynamic enhanced MRI enables clear visualization of lesion morphology and surrounding vascular shadow, and quantitative analysis of vessel structure and function by injecting contrast agent to observe its diffusion pattern among capillaries and lesions and then reflecting the enhancement characteristics of tumor lesions and calculating parameters such as *K*^trans^, *K*_ep_, and *V*_e_. Compared with pathological findings, dynamic enhanced MRI also showed high diagnostic efficacy, but considering the high cost of this method, clinical promotion should be carried out based on local medical and economic levels.

### 4.3. Diagnostic Value of Combining Dynamic Enhanced MRI with Ultrasonic DOT in Early Breast Cancer

After respectively comparing the diagnostic results of dynamic enhanced MRI and ultrasonic DOT with the pathologic findings, it was believed that combined diagnosis had significantly higher diagnosis accuracy rate, sensitivity, specificity, PPV and NPV than the dynamic enhanced MRI and ultrasonic DOT diagnosis alone (*P* < 0.05); by further analyzing the efficacy of the two diagnosis modalities in diagnosing early breast cancer by ROC curves, the result was combined diagnosis > dynamic enhanced MRI > ultrasonic DOT. Ultrasonic DOT, which effectively combines optical technology with acoustic technology, and can directly obtain the functional information of tissues with convenient operation and no need for intravenous contrast. In addition, it can also carry out comprehensive evaluation of structural information and functional information of lesions, which is a beneficial supplement to the field of modern medical imaging relying solely on morphology to tumor diagnosis, and in particular, presents a potential warning value in atypical hyperplasia. Dynamic enhanced MRI has good accuracy, sensitivity and specificity for breast disease. However, it is complex, expensive, and time-consuming, and requires venography to obtain accurate information of lesions, so it is not recommended as the first choice for early breast cancer screening, but can be used as an important supplement to breast cancer diagnosis and effectively combined with ultrasonic DOT to increase the rate of clinical diagnosis of breast cancer.

The shortcomings of this study: (1) It was a retrospective analysis study, thus there may be selection bias and recall bias; patients' data were limited; and relative risks could not be analyzed directly. (2) The sample size was small, so the examination efficacy may not be achieved.

In conclusion, both dynamic enhanced MRI and ultrasonic DOT have high diagnostic values for early breast cancer, in which dynamic enhanced MRI obtains results closer to pathologic findings, and has diagnostic efficacy higher than that of ultrasonic DOT. However, the combination of the two can significantly improve the diagnostic accuracy of early breast cancer and has higher diagnostic value, so it is suggested that ultrasonic DOT should be considered as the primary screening method for early breast cancer in the clinic, supplemented by dynamic enhanced MRI.

## Figures and Tables

**Figure 1:** ROC curve.

**Table 1:** Between-group comparison of patients' general data.

Observation indicator	Benign lesion group (*n* = 50)	Breast cancer group (*n* = 60)	*X* ^2^/*t*	*P*

Age (years)	49.75 ± 7.22	50.13 ± 6.94	0.281	0.779
BMI (kg/m^2^)	21.40 ± 3.21	21.15 ± 3.16	0.410	0.623
Tumor diameter (cm)	0.68 ± 0.17	0.69 ± 0.15	0.328	0.748
*Histological grade*				
I	6 (12.00)	3 (5.00)	1.779	0.182
II	29 (58.00)	36 (60.00)	0.045	0.832
III	15 (30.00)	21 (35.00)	0.310	0.578

*Molecular typing*				
Luminal A	10 (20.00)	14 (23.33)	0.178	0.673
Luminal B	26 (52.00)	26 (43.34)	0.822	0.365
HER-2 overexpression	4 (8.00)	6 (10.00)	0.132	0.716
Triple negative	10 (20.00)	14 (23.33)	0.178	0.673

*Number of masses*				
Single mass	27 (54.00)	35 (58.33)	0.208	0.648
2	21 (42.00)	22 (36.67)	0.326	0.568
≥3	2 (4.00)	3 (5.00)	0.063	0.802

**Table 2:** DWI image characteristics.

Group	Irregular shape	Increased vascular shadow	Obscure boundary	Spicule sign	Heterogeneous enhancement

Benign lesion group (*n* = 50)	10 (20.00)	14 (28.00)	8 (13.00)	6 (12.00)	9 (18.00)
Breast cancer group (*n* = 60)	31 (51.67)	46 (76.67)	44 (73.33)	27 (45.00)	33 (55.00)
*X* ^2^	11.697	26.053	35.966	14.123	15.818
*P*	0.001	<0.001	<0.001	<0.001	<0.001

**Table 3:** Comparison of dynamic enhanced MRI parameters.

Group	*K* ^trans^ (min)	*K*_ep_ (min)	*V*_e_

Benign lesion group (*n* = 50)	0.44 ± 0.08	0.63 ± 0.15	0.69 ± 0.20
Breast cancer group (*n* = 60)	0.59 ± 0.16	0.94 ± 0.23	1.07 ± 0.22
*t*	6.028	8.186	9.398
*P*	<0.001	<0.001	<0.001

**Table 4:** Between-group comparison of THC values.

Group	*n*	THC (*μ*mol/L)

Benign lesion group	50	135.64 ± 16.90
Breast cancer group	60	205.42 ± 18.15
*t*		20.713
*P*		<0.001

**Table 5:** Comparison with pathologic findings.

Pathologic finding	*n*	Combined diagnosis		Dynamic enhanced MRI		Ultrasonic DOT	
		+	−	+	−	+	−

+	60	57	3	54	6	50	10
−	50	5	45	8	42	11	39

**Table 6:** Analysis on diagnostic value of single diagnosis and combined diagnosis for breast cancer (%).

Examination indicator	Accuracy rate	Sensitivity	Specificity	PPV	NPV

Combined diagnosis	92.73	95.00	90.00	91.94	93.75
Dynamic enhanced MRI	87.27	90.00	84.00	87.10	87.50
Ultrasonic DOT	80.91	83.33	78.00	91.97	79.59

**Table 7:** Area under curve.

Test result variable	Area	SE^a^	Asymp. sig.^b^	Asymp. 95%CI

Combined diagnosis	0.925	0.030	0.000	0.867–0.983
Dynamic enhanced MRI	0.870	0.038	0.000	0.796–0.944
Ultrasonic DOT	0.807	0.044	0.000	0.720–0.893

^a^∂*G*(*x*)/∂*y* < 0 under nonparametric assumptions. ^b^Null hypothesis: solid area = 0.5;

## Data Availability

Data to support the findings of this study is available on reasonable request from the corresponding author.
